The article "Total Glucosides of Peony Protect Cardiomyocytes against Oxidative Stress and Inflammation by Reversing Mitochondrial Dynamics and Bioenergetics" was retracted in 2023. Reasons: signs of a paper mill; suspected computer-generated content; unreliable results or conclusions; concerns about the data.

# Total Glucosides of Peony Protect Cardiomyocytes against Oxidative Stress and Inflammation by Reversing Mitochondrial Dynamics and Bioenergetics

**DOI:** 10.1155/2020/6632413

**Published:** 2020-11-25

**Authors:** Mengmeng Wang, Qiang Li, Ying Zhang, Hao Liu

**Affiliations:** ^1^Department of Rheumatism and Immunology, Tianjin First Central hospital, Tianjin, China; ^2^Department of Pharmacy, Tianjin Union Medical Center, Tianjin, China; ^3^Department of Cardiology, Chinese PLA General Hospital, Beijing, China; ^4^Department of Pharmacy, Nankai University, Tianjin, China

## Abstract

Total glucosides of peony (TGP) are used to treat rheumatoid arthritis and systemic lupus erythematosus. We explored the protective effects of TGP on cardiomyocyte oxidative stress and inflammation in the presence of hydrogen peroxide by focusing on mitochondrial dynamics and bioenergetics. Our study demonstrated that hydrogen peroxide significantly repressed cardiomyocyte viability and promoted cell apoptosis through induction of the mitochondrial death pathway. TGP treatment sustained cardiomyocyte viability, reduced cardiomyocyte apoptosis, and decreased inflammation and oxidative stress. Molecular investigation indicated that hydrogen peroxide caused mitochondrial dynamics disruption and bioenergetics reduction in cardiomyocytes, but this alteration could be normalized by TGP. We found that disruption of mitochondrial dynamics abolished the regulatory effects of TGP on mitochondrial bioenergetics; TGP modulated mitochondrial dynamics through the AMP-activated protein kinase (AMPK) pathway; and inhibition of AMPK alleviated the protective effects of TGP on mitochondria. Our results showed that TGP treatment reduces cardiomyocyte oxidative stress and inflammation in the presence of hydrogen peroxide by correcting mitochondrial dynamics and enhancing mitochondrial bioenergetics. Additionally, the regulatory effects of TGP on mitochondrial function seem to be mediated through the AMPK pathway. These findings are promising for myocardial injury in patients with rheumatoid arthritis and systemic lupus erythematosus.

## 1. Introduction

Total glucosides of peony (TGP) are used to treat rheumatoid arthritis and systemic lupus erythematosus [1] as well as hepatitis, dysmenorrhea, muscle cramps, and spasms. The active components of TGP include monoterpene glycosides, galloyl glucoses, and phenolic compounds [2]. In long-term clinical use, TGP have therapeutic effects and no severe side effects [3–5]. Anti-inflammatory activity has been identified as the primary molecular mechanism underlying TGP [6]. In animal studies, TGP administration has been shown to impair inflammation cell activation and recruitment [4]. Inflammation-related signaling pathways such as NF-*κ*B [7] and home oxygenase-1 are also regulated by TGP [8]. TGP has also been used as an antioxidant to decrease reactive oxygen species (ROS) production and oxidative stress [9, 10]. TGP treatment activates the Nrf2 signaling pathway, contributing to the transcriptional upregulation of anti-oxidative factors such as superoxide dismutase (SOD) and glutathione (GSH) [11, 12]. The anti-inflammatory and anti-oxidative properties of TGP make it a promising option for the treatment of diabetic nephropathy [13], kidney injury [14], fatty liver disease [15], and pulmonary arterial hypertension [16]. However, the regulatory effects of TGP on cardiomyocyte (patho)physiological responses have not been fully explored.

The article "Total Glucosides of Peony Protect Cardiomyocytes against Oxidative Stress and Inflammation by Reversing Mitochondrial Dynamics and Bioenergetics" was retracted in 2023. Reasons: signs of a paper mill; suspected computer-generated content; unreliable results or conclusions; concerns about the data.

Cardiomyocyte oxidative stress and inflammation are risk factors for the development of cardiovascular diseases such as ischemic heart disorder, myocardial ischemia-reperfusion injury, diabetic cardiomyopathy, myocardial fibrosis, and hypertension [17–20]. At the molecular level, cardiomyocytes contain abundant mitochondria, which generate adenosine triphosphate (ATP) to mediate cardiomyocyte contractility [21, 22]. However, damaged mitochondria cannot transfer electrons, which subsequently convert into ROS [23]. Excessive ROS production is associated with cardiomyocyte oxidative stress [24, 25] resulting in cardiomyocyte dysfunction or death. Oxidative stress is also followed by increased inflammation, which is used to repair damaged myocardium or remove dead cardiomyocytes [26–28]. However, uncontrolled inflammation promotes myocardial edema, induces the accumulation of inflammation cells, and augments cytokine release, a process that attends cardiac fibroblast proliferation and collagen deposition [29, 30]. These pathological alterations have been observed in postinfarction cardiac injury, heart failure, and diabetic cardiomyopathy [31, 32]. In this study, we verified whether TGP can attenuate mitochondrial damage and thus repress oxidative stress and inflammation in cardiomyocytes.

Mitochondria regulate cardiomyocyte oxidative stress and inflammation [33, 34]. Impaired mitochondrial metabolism is followed by ROS production and inflammation. Several mechanisms have been proposed to explain impaired mitochondrial metabolism, such as mitochondrial complex inactivation and mitochondrial metabolism switch from oxidative phosphorylation to glycolysis [35, 36]. It is necessary to explore whether TGP has the ability to normalize mitochondrial metabolism in cardiomyocytes. Recent studies have reported that disruption of mitochondrial dynamics, an alteration of mitochondrial morphology, functions upstream of mitochondrial metabolism switching [37, 38]. However, it is unclear whether TGP affects cardiomyocyte function and viability by affecting mitochondrial dynamics and bioenergetics. This study explored the protective effect of TGP on cardiomyocyte oxidative stress and inflammation by focusing on mitochondrial dynamics and bioenergetics.

The article "Total Glucosides of Peony Protect Cardiomyocytes against Oxidative Stress and Inflammation by Reversing Mitochondrial Dynamics and Bioenergetics" was retracted in 2023. Reasons: signs of a paper mill; suspected computer-generated content; unreliable results or conclusions; concerns about the data.

## 2. Materials and Methods

### 2.1. Cell Cultures

The H9C2 cardiomyocyte cell line was purchased from the Beijing Union Cell Resource Center. H9C2 cells were cultivated in DMEM (Gibco, USA) medium supplemented with 15% fetal bovine serum (FBS) (modified, Gibco, USA), 100 IU/mL penicillin, and 100 *μ*g/mL streptomycin in a 5% CO_2_ incubator at 37°C. Hydrogen peroxide (0.3 mM) was added to the medium to induce oxidative stress. TGP purchased from Sigma was added to the medium at a final concentration of 300 mol/L for 24 hours before hydrogen peroxide treatment [39].

### 2.2. Mitochondrial Membrane Potential and Mitochondrial ROS Detection

To observe mitochondrial membrane potential, we added 5 mg/L JC-1 staining buffer to the cardiomyocyte medium for 30 min in the dark. Cells were then washed with PBS to remove free JC-1. Using a multifunctional microplate reader, we set the excitation light to 490 nm and the emission light to 530 nm to detect JC-1 monomers, and we set the excitation light to 525 nm and the emission light to 590 nm to detect JC-1 polymers [40]. We used the ratio of red to green fluorescence to measure the degree of mitochondrial membrane potential depolarization.

### 2.3. Determination of the Opening Level of Mitochondrial Permeability Transition Pore (mPTP)

After cells were collected, we turned on the multifunctional microplate reader in advanced mode and set the temperature to 25°C and the wavelength to 540 nm (reading starting at 10 min and every 30 sec until 30 min); before initiating the program, we set it to zero. Next, we pipetted 20 *μ*L of cell suspension concentrated at 10 *μ*g/*μ*L into the corresponding wells of a 96-well plate. We then added 170 *μ*L of buffer Reagent A, mixed it well, and immediately placed it into the microplate reader (wavelength, 540 nm) to read the absorbance value at A540 [41]. After the samples stood at room temperature for 1 min, we reread the absorbance value at A540. At that point, the recorded initial A540 value was 0 min. Next, we added 10 *μ*L of Reagent B and mixed it well [42]. We immediately put the plate into the multifunctional microplate reader (wavelength, 540 nm) and dynamically recorded the change values of the actual absorbance value for 10 min. Finally, we calculated the ratio of absorbance (A540/initial A540).

The article "Total Glucosides of Peony Protect Cardiomyocytes against Oxidative Stress and Inflammation by Reversing Mitochondrial Dynamics and Bioenergetics" was retracted in 2023. Reasons: signs of a paper mill; suspected computer-generated content; unreliable results or conclusions; concerns about the data.

### 2.4. Detection of Mitochondrial Morphology

Mitochondrial morphology was evaluated in H9c2 cells that were incubated with a 100 nM MitoTracker Green probe (Thermo Fisher Scientific, Waltham, MA, USA) for 30 min at 37°C. Images were acquired using a confocal laser scanning microscope (FV 1000, Olympus, Tokyo, Japan) [43]. The percentage of cells with fragmented mitochondria (small and round) was determined.

### 2.5. Immunofluorescence

After fixation with 4% paraformaldehyde, the cells were permeated with 0.5% Triton X-100 for 15 min, blocked with 10% donkey serum for 30 min, and stained with a TdT-mediated dUTP Nick-End Labeling (TUNEL) Kit (C1086, Beyotime, Shanghai, China) according to the manufacturer's instructions. The slides or cells were incubated with the TUNEL cocktail for 1 h. After washing with PBS 3 times, the slides or cells were incubated with sarcomeric *α* actinin and LC3B antibodies overnight at 4°C [44]. The next day, the slides or cells were incubated with secondary antibodies, wheat germ agglutinin (WGA), and 4',6-diamidino-2-phenylindole (DAPI) for 30 min. Three researchers who were blind to the sample identified quantified TUNEL by either manual counting or digital thresholding. This included image segmentation and the creation of a binary image from grayscale [45]. We analyzed the converted binary images using the ImageJ software (NIH, Bethesda, MA, USA; Laboratory for Optical and Computational Instrumentation, University of Wisconsin-Madison, WI, USA).

### 2.6. Mitochondrial ROS Assay

The production of mitochondrial ROS in the H9C2 cells was detected using a MitoSOX red mitochondrial superoxide indicator (Molecular Probes, USA). After various treatments, H9C2 cells were incubated with MitoSOX (10 *μ*M) and stained in the dark at 37°C for 30 min. The fluorescent image was then captured by a fluorescence microscope, and the fluorescence intensity was calculated using the ImageJ software [46].

### 2.7. Measurement of Caspase-3 Activity

Caspase-3 activity was determined by measuring the generation of the fluorogenic cleavage product methylcoumarylamide using a Caspase-3 Activity Assay Kit (Beyotime, Shanghai, China) according to the manufacturer's instructions [47]. H9C2 cells were briefly homogenized in an ice-cold buffer and then centrifuged at 1000 *g* for 5 min. After centrifugation, the supernatant was transferred to a new tube for caspase-3 activity testing. Fluorescence from a 100 *μ*L sample was assayed in fluorescent spectrophotometry with 100 *μ*L of detection buffer and then normalized by protein concentration [48].

### 2.8. siRNA Knockdown

Drp1 siRNAs were purchased from Dharmacon (OnTarget-Plus Smart Pool). Cells were washed and incubated with 20 nM siRNA in OptiMEM media (Life Technologies #31985070) supplemented with 1 : 50 Oligofectamine (Life Technologies #12252011) for 5 hours. Cells were then washed with 1X PBS and incubated overnight with DMEM supplemented with 30% FBS and no antibiotics [49]. The next day, the cells were washed with 1X PBS and used for the experiments.

The article "Total Glucosides of Peony Protect Cardiomyocytes against Oxidative Stress and Inflammation by Reversing Mitochondrial Dynamics and Bioenergetics" was retracted in 2023. Reasons: signs of a paper mill; suspected computer-generated content; unreliable results or conclusions; concerns about the data.

### 2.9. Measurement of Inflammation Factors Levels

The levels of MCP1 and TNF*α* were measured using ELISA kits following the protocols provided by the manufacturer (R&D Systems, Inc. MN) [50].

### 2.10. SDS/PAGE and Immunoblotting

Samples were briefly heated to 50°C for 5 min in beta-mercaptoethanol 4x loading buffer and then run on 4-20% Criterion precast gels (Bio-Rad, CA) in 0.1% SDS Tris glycine running buffer. The SDS-PAGE-resolved proteins were transferred to iBlot stacks with regular PVDF membranes using the Life Technologies iBlot 2 system. Nonspecific binding sites were blocked with 5% nonfat dry milk in PBS-T (3 mM KH_2_PO_4_, 10 mM Na_2_HPO_4_, 150 mM NaCl, 0.1% Tween 20, and pH 7.2-7.4) for 30 min at room temperature. Membranes were then incubated with specific primary antibodies diluted in 5% nonfat dry milk in PBS-T overnight at 4°C. After washing 3 times for 10 min, membranes were incubated with horseradish peroxidase conjugated secondary antibodies diluted in 5% nonfat dry milk in PBS-T for 1 h. After washing 3 times for 10 min, protein-antibody reactions were detected by SuperSignal chemiluminescence (Pierce Biotechnology Inc., Rockford, IL) and imaged using the Image Lab software 5 (Bio-Rad). Protein densities were measured using the Image Lab software 5 [51]. For Western blot tests of total cell extraction, a classic Bradford protein concentration assay was used for protein quantification; 30-50 *μ*g of protein was suspended in 4x Laemmli buffer to load a final volume of 30 *μ*L. Samples were not reduced for Western blot tests of biotinylation. Western blots against the NaV 1.5 protein were performed, and then the membranes were stripped and reblotted with conjugated streptavidin HRP [52].

### 2.11. Measurement of Lactate Product and Adenosine Triphosphate (ATP) Level

The L-Lactate Assay Kit and the ATP Assay Kit (both from Sigma-Aldrich, Taufkirchen, Germany) were used according to the manufacturer's instructions to determine the levels of lactate product and ATP [53].

### 2.12. Real-Time Polymerase Chain Reaction (PCR)

Total RNA was extracted from samples using TRIzol Reagent (Thermo Fisher) and digested with DNase I (Invitrogen) to eliminate genomic DNA. cDNA was synthetized using the SuperScript III First-Strand Synthesis System for RT-PCR (Invitrogen) according to the manufacturer's instructions [54]. Real-time PCR was performed using the QuantiFast SYBR Green PCR Kit (Qiagen) and the StepOnePlus Real-Time PCR System (Applied Biosystems). Ct values were normalized with respect to *β*-actin. Fold change was calculated with respect to sham vehicle [55].

The article "Total Glucosides of Peony Protect Cardiomyocytes against Oxidative Stress and Inflammation by Reversing Mitochondrial Dynamics and Bioenergetics" was retracted in 2023. Reasons: signs of a paper mill; suspected computer-generated content; unreliable results or conclusions; concerns about the data.

### 2.13. Statistics

All data are expressed as mean ± SEM. Statistical differences were measured using a paired or unpaired two-sided Student's *t*-test and one-way ANOVA with Bonferroni or Dunnett corrections for multiple comparisons when appropriate. A value of *P* < 0.05 was considered statistically significant. Data analysis was performed using the GraphPad Prism software, version 7 (GraphPad Software, San Diego, CA).

## 3. Results

### 3.1. TGP Administration Significantly Reduces Cardiomyocyte Apoptosis and Inflammation in the Presence of Hydrogen Peroxide

In this study, cardiomyocytes were pretreated with TGP and then cultured with hydrogen peroxide to induce oxidative stress and inflammation. Cardiomyocyte viability was then determined using a CCK-8 assay. Compared to the control group, hydrogen peroxide administration significantly reduced cell viability, but this alteration could be attenuated by the TGP treatment (Figure 1(a)). Western blots were used to analyze the alteration of apoptosis-related proteins. As shown in Figures 1(b)–1(e), compared to the control group, the expression of caspase-9, Bax, and Bad was elevated by hydrogen peroxide, but this trend could be inhibited by TGP pretreatment. This data indicates that cardiomyocyte viability can be reversed by TGP in the presence of hydrogen peroxide.

Next, we analyzed the alteration of inflammation factors in response to TGP treatment. The levels of proinflammatory factors such as TNF*α* and MCP1 were upregulated in response to hydrogen peroxide treatment (Figures 1(f) and 1(g)). However, TGP exerts anti-inflammatory action to prevent the activation of proinflammatory factors (Figures 1(f) and 1(g)). These results indicate that TGP administration reduces cardiomyocyte apoptosis and inflammation in the presence of hydrogen peroxide.

### 3.2. Cardiomyocyte Oxidative Stress Is Attenuated by TGP

To understand the alteration of oxidative stress in TGP-treated cardiomyocytes, a mitochondrial ROS probe was used. As shown in Figures 2(a) and 2(b), compared to the control group, the levels of mitochondrial ROS were upregulated in response to hydrogen peroxide treatment. TGP treatment repressed the production of mitochondrial ROS in cardiomyocytes (Figures 2(a) and 2(b)), supporting the antioxidative effects of TGP on hydrogen peroxide-treated cardiomyocytes. Decreased ROS production results from two molecular mechanisms; one is driven by the enhanced antioxidative action of TGP, and the other is involved in decreased ROS production in mitochondria. Therefore, we analyzed the alteration of antioxidative factors in response to TGP treatment. As shown in Figures 2(c)–2(e), compared to the control group, the activity of antioxidative enzymes such as SOD, GSH, and glutathione peroxidase (GPX) was reduced by hydrogen peroxide, but this alteration could be reversed by TGP, suggesting that TGP treatment enhanced the anti-oxidative defense system in hydrogen peroxide-treated cardiomyocytes. We also analyzed the regulatory effect of TGP on mitochondrial complexes I and III, which are the primary sites for ROS production. As shown in Figures 2(f) and 2(g), compared to the control group, the activity of complex I/III was downregulated by hydrogen peroxide in cardiomyocytes. Decreased complex I/III cannot capture electrons, resulting in ROS production [28]. In comparison, TGP treatment drastically improved the activities of complex I/III in hydrogen peroxide-treated cardiomyocytes (Figures 2(f) and 2(g)). These results indicate that TGP-afforded antioxidative action is mediated by increased antioxidative stress and decreased mitochondrial ROS production.

The article "Total Glucosides of Peony Protect Cardiomyocytes against Oxidative Stress and Inflammation by Reversing Mitochondrial Dynamics and Bioenergetics" was retracted in 2023. Reasons: signs of a paper mill; suspected computer-generated content; unreliable results or conclusions; concerns about the data.

### 3.3. Mitochondrial Dynamics and Bioenergetics Are Normalized by TGP

Mitochondrial dynamics and bioenergetics are closely associated with cardiomyocyte damage, especially oxidative stress and inflammation [37]. Thus, we analyzed the regulatory effects of TGP on mitochondrial dynamics and bioenergetics. First, mitochondrial membrane potential, the marker of mitochondrial bioenergetics, was stained by JC-1. Hydrogen peroxide treatment significantly reduced mitochondrial membrane potential (Figures 3(a) and 3(b)), represented by decreased red fluorescence and increased green fluorescence. TGP treatment stabilized mitochondrial membrane potential in the presence of hydrogen peroxide. Cellular ATP production was also derived from mitochondrial bioenergetics. As shown in Figure 3(c), compared to the control group, hydrogen peroxide reduced the ATP content, whereas TGP favored ATP synthesis in cardiomyocytes. These results indicate that mitochondrial bioenergetics can be stabilized by TGP in hydrogen peroxide-treated cardiomyocytes.

Immunofluorescence also demonstrated a fragmented mitochondrial network in hydrogen peroxide-treated cardiomyocytes (Figures 3(d)–3(f)), suggesting a disruption in mitochondrial dynamics. RNA analysis demonstrated that mitochondrial fission genes were upregulated, whereas the transcription of mitochondrial fusion genes was drastically repressed in hydrogen peroxide-treated cardiomyocytes (Figures 3(g) and 3(h)). In TGP-treated cardiomyocytes, the normal mitochondrial network was sustained, and the ratio of fragmented mitochondria was reduced, followed by normalization of mitochondrial dynamics. To understand whether mitochondrial dynamics function upstream of bioenergetics, an adenovirus-mediated Drp1 overexpression assay was conducted. In Drp1-overexpressed cardiomyocytes, TGP failed to sustain ATP production (Figure 3(i)), suggesting that TGP regulated bioenergetics by normalizing mitochondrial dynamics.

The article "Total Glucosides of Peony Protect Cardiomyocytes against Oxidative Stress and Inflammation by Reversing Mitochondrial Dynamics and Bioenergetics" was retracted in 2023. Reasons: signs of a paper mill; suspected computer-generated content; unreliable results or conclusions; concerns about the data.

### 3.4. Induction of Mitochondrial Fission Abolishes the Beneficial Effects of TGP on Mitochondrial Function and Cardiomyocyte Viability

To understand whether mitochondrial dynamics are required for TGP-sustained mitochondrial function and cardiomyocyte viability, Drp1-mediated mitochondrial fission was induced in TGP-treated cardiomyocytes. Mitochondrial function and cardiomyocyte viability were then remeasured. As shown in Figures 4(a) and 4(b), compared to the control group, although TGP repressed mitochondrial ROS production, this effect was abolished by Drp1 overexpression. In Drp1-overexpressed cardiomyocytes, TGP failed to sustain mitochondrial potential in the presence of hydrogen peroxide (Figures 4(c) and 4(d)). These results indicate that TGP controlled mitochondrial function by correcting disrupted mitochondrial dynamics.

In addition, hydrogen peroxide-mediated cardiomyocyte viability reduction could be reversed by TGP, but this protective effect was undetectable in Drp1-overexpressed cardiomyocytes. In accordance with this finding, hydrogen peroxide elevated the activity of caspase-3, but this alteration could be repressed by TGP (Figure 4(e)). The antiapoptotic action of TGP was blocked by Drp1 overexpression, suggesting that TGP protects cardiomyocyte viability and mitochondrial fusion by preserving mitochondrial dynamics.

### 3.5. TGP Maintains Mitochondrial Dynamics through the AMPK Pathway

Previous studies have reported a link between the AMP-activated protein kinase (AMPK) pathway and mitochondrial dynamics [56]. In diabetic cardiomyopathy, AMPK activation is followed by decreased mitochondrial fission and increased mitochondrial fusion through the inhibition of Drp1 activation. Ample evidence indicates the promotive role of TGP in inducing AMPK activation. Therefore, we investigated whether TGP modulated mitochondrial dynamics through the AMPK pathway. First, Western blots were used to observe the alteration of AMPK in response to hydrogen peroxide or TGP treatment. As shown in Figures 5(a) and 5(b), compared to the control group, AMPK expression was significantly reduced, followed by a decline in AMPK activity (Figure 5(c)). TGP treatment elevated AMPK expression (Figures 5(a) and 5(b)) and improved AMPK activity (Figure 5(c)), suggesting that TGP can correct hydrogen peroxide-mediated AMPK inhibition. To understand whether TGP modulates mitochondrial dynamics through AMPK, compound C, an AMPK pathway inhibitor, was added to TGP-treated cardiomyocytes. Mitochondrial dynamics were then reanalyzed. As shown in Figures 5(d) and 5(e), hydrogen peroxide upregulated the transcription of mitochondrial fission-related genes, but this phenotypic alteration could be attenuated by TGP. Inhibition of the AMPK pathway abolished the regulatory effect of TGP on mitochondrial fission (Figures 5(d) and 5(e)). Similarly, mitochondrial fusion-related genes were drastically upregulated by TGP in the presence of hydrogen peroxide, but this effect was not seen in cardiomyocytes treated with compound C (Figures 5(d) and 5(e)). These results indicate that the AMPK pathway is involved in TGP-regulated mitochondrial dynamics.

The article "Total Glucosides of Peony Protect Cardiomyocytes against Oxidative Stress and Inflammation by Reversing Mitochondrial Dynamics and Bioenergetics" was retracted in 2023. Reasons: signs of a paper mill; suspected computer-generated content; unreliable results or conclusions; concerns about the data.

## 4. Discussion

In this study, we explored the cardioprotective effects of TGP on cardiomyocyte oxidative stress and inflammation by focusing on mitochondrial dynamics and bioenergetics. After exposure to hydrogen peroxide, cardiomyocyte viability was reduced, but the apoptosis rate was increased. Mitochondria-mediated apoptosis has been regarded as the primary reason for the initiation of cardiomyocyte death. TGP treatment significantly reduced cardiomyocyte death by blocking mitochondrial apoptosis. We also observed the antioxidative and anti-inflammatory actions of TGP on hydrogen peroxide-treated cardiomyocytes. At the molecular level, TGP upregulated the activities of antioxidative factors and inhibited the formation of mitochondrial ROS, resulting in inhibition of oxidative stress in cardiomyocytes. Additionally, TGP administration was associated with a drop in the transcription of proinflammatory genes. Molecular investigation demonstrated that TGP modulated mitochondrial function by correcting mitochondrial dynamics and improving mitochondrial bioenergetics. Disruption of mitochondrial dynamics abolished the protective effects of TGP on mitochondrial bioenergetics, suggesting that mitochondrial dynamics function upstream of bioenergetics. Finally, we observed that TGP modulated mitochondrial dynamics and bioenergetics through the AMPK pathway. Our results showed that TGP played a cardioprotective role in cardiomyocyte oxidative stress and inflammation by normalizing mitochondrial dynamics and improving mitochondrial bioenergetics. This finding supports the use of TGP in regulating cardiomyocyte viability, especially in rheumatoid arthritis.

The article "Total Glucosides of Peony Protect Cardiomyocytes against Oxidative Stress and Inflammation by Reversing Mitochondrial Dynamics and Bioenergetics" was retracted in 2023. Reasons: signs of a paper mill; suspected computer-generated content; unreliable results or conclusions; concerns about the data.

Several studies have reported the antioxidative, anti-inflammatory, and antiproliferative properties of TGP. For example, in a mice model of constipation and intestinal inflammation, TGP significantly reduced the symptoms and improved the prognosis [57]. TGP also alleviates cerebral ischemia-reperfusion injury by modulating the inflammation response [58]. At the molecular level, Toll-like receptor-2 [59], TNF receptor-associated factor [59], NF-*κ*B [59], microphthalmia-associated transcription factor (MITF) [60], and tyrosinase-related protein 1 (TRP-1) [60] have been regarded as the downstream targets of TGP. In this study, we found that TNF*α* and MCP1 could be reduced by TGP in hydrogen peroxide-treated cardiomyocytes, confirming the anti-inflammatory action of TGP. Additionally, we found that the levels of cellular antioxidative factors were significantly elevated by TGP. Mitochondrial complex activity was also normalized by TGP, resulting in a decline in the production of mitochondrial ROS in cardiomyocytes. These findings suggest that TGP regulates oxidative stress by affecting ROS-related signaling pathways, such as the Nrf2/ARE axis [61] or the PKC*δ*/NF-*κ*B pathway [62].

Mitochondrial dynamics are alterations of mitochondrial shape and size and include mitochondrial fission and fusion [63–66]. Increased mitochondrial fission and decreased mitochondrial fusion are apoptotic signals for cardiomyocytes under stressful conditions, including but not limited to cardiac ischemia-reperfusion injury, diabetic cardiomyopathy, heart failure, and sepsis-related myocardial damage [21, 27]. Disruption of mitochondrial dynamics is followed by mitochondrial fragmentation with low mitochondrial membrane potential and increased mitochondrial ROS production [67–69]. In this study, we observed that disruption of mitochondrial dynamics is followed by mitochondrial damage and cardiomyocyte death. TGP treatment has the ability to reverse mitochondrial dynamics and thus promote mitochondrial bioenergetics, leading to increased cellular ATP production. Previous studies have reported the regulatory effects of TGP on mitochondria. In retinal pigment epithelial cells, TGP attenuates oxidative stress-related mitochondrial dynamics by activating the CaMKII/AMPK pathway [9]. In streptozotocin-induced cognitive impairment in mice, TGP treatment sustains mitochondrial membrane potential, promotes ATP synthesis, and blocks mitochondrial apoptosis [70]. These results suggest that the molecular mechanism underlying TGP-mediated cardioprotection and mitochondria may be the potential targets of TGP.

Our results showed that TGP treatment improves cardiomyocyte oxidative stress and inflammation in the presence of hydrogen peroxide by correcting mitochondrial dynamics and enhancing mitochondrial bioenergetics. Additionally, the regulatory effects of TGP on mitochondrial function seem to be mediated through the AMPK pathway. These findings are promising for the treatment of myocardial injury in patients with rheumatoid arthritis and systemic lupus erythematosus.

The article "Total Glucosides of Peony Protect Cardiomyocytes against Oxidative Stress and Inflammation by Reversing Mitochondrial Dynamics and Bioenergetics" was retracted in 2023. Reasons: signs of a paper mill; suspected computer-generated content; unreliable results or conclusions; concerns about the data.

## Figures and Tables

**Figure 1:** TGP treatment attenuates cardiomyocyte apoptosis and inflammation induced by hydrogen peroxide. (a) Cardiomyocyte cell viability was determined using a CCK-8 assay. (b–e) Western blots were used to observe the alterations of caspase-9, Bax, and Bad in cardiomyocytes treated with TGP in the presence of hydrogen peroxide. (f, g) RNA was isolated from cardiomyocytes, then the transcription of MCP1*α* and MCP1 was analyzed using qPCR. ∗*p* < 0.05.

**Figure 2:** Cardiomyocyte oxidative stress is attenuated by TGP. (a, b) Mitochondrial ROS was determined through immunofluorescence in response to TGP treatment. (c–e) The levels of antioxidative stress, including SOD, GSH, and GXP, were measured by ELISA. (f, g) The activity of mitochondrial complexes I and III was determined by ELISA. ∗*p* < 0.05.

**Figure 3:** Mitochondrial dynamics and bioenergetics are normalized by TGP. (a, b) Mitochondrial membrane potential was observed using a JC-1 probe. (c) ATP production was measured by ELISA in cardiomyocytes treated with TGP. (d–f) Mitochondrial morphology was observed through immunofluorescence. (g, h) RNA was isolated from cardiomyocytes, then the transcription of MCP1*α* and MCP1 was analyzed using qPCR. (i) ATP production was determined by ELISA in cardiomyocytes transfected with Drp1 adenovirus. ∗*p* < 0.05.

**Figure 4:** Induction of mitochondrial fission abolishes the beneficial effects of TGP on mitochondrial function and cardiomyocyte viability. (a, b) Mitochondrial ROS was determined by immunofluorescence in response to TGP treatment. Drp1 adenovirus was transfected into cardiomyocytes to overexpress Drp1. (c, d) Mitochondrial membrane potential was observed using a JC-1 probe. (e) ELISA was used to observe the alteration of caspase-3. ∗*p* < 0.05.

**Figure 5:** TGP maintains mitochondrial dynamics through the AMPK pathway. (a, b) Western blots were used to observe the alteration of AMPK in cardiomyocytes treated with TGP in the presence of hydrogen peroxide. Drp1 adenovirus was transfected into cardiomyocytes to overexpress Drp1. (c) ELISA was used to evaluate the activity of AMPK. (d, e) RNA was isolated from cardiomyocytes, then the transcription of MCP1*α* and MCP1 was analyzed using qPCR. Compound C was used to inhibit the activity of AMPK. ∗*p* < 0.05.

The article "Total Glucosides of Peony Protect Cardiomyocytes against Oxidative Stress and Inflammation by Reversing Mitochondrial Dynamics and Bioenergetics" was retracted in 2023. Reasons: signs of a paper mill; suspected computer-generated content; unreliable results or conclusions; concerns about the data.

## Data Availability

All data generated or analyzed during this study are included in this article.
